RETRACTED

# MicroRNA-326 Functions as a Tumor Suppressor in Breast Cancer by Targeting ErbB/PI3K Signaling Pathway

**DOI:** 10.3389/fonc.2019.00653

**Published:** 2019-07-30

**Authors:** Zahra Ghaemi, Bahram Mohammad Soltani, Seyed Javad Mowla

**Affiliations:** Department of Genetics, Faculty of Biological Sciences, Tarbiat Modares University, Tehran, Iran

**Keywords:** ErbB/PI3K signaling pathway, miR-326, breast cancer, tumor suppressor, microRNA

## Abstract

Breast cancer represents the most common malignancy in women worldwide and the ErbB/PI3K pathway has been found to play a crucial role in regulation of the cancer cell growth. MicroRNAs have been implicated in regulating diverse cellular pathways and therefore, understanding the link between the regulatory microRNAs and the ErbB/PI3K signaling pathway could potentially be helpful for breast cancer prevention and treatment. The aim of this study is to examine the regulatory effect of miR-326 on ErbB/PI3K signaling pathway in breast cancer development and progression. The results of qRT-PCR, RNA seq, and array data indicated that miR-326 was remarkably down-regulated in breast tumor tissues and correlated with poor survival outcome. Importantly, very low levels of miR-326 expression were found in aggressive breast cells compared to less-aggressive cell types. Mechanistically, a gene network including *EGFR, ErbB2, ErbB3, AKT1, AKT2*, and *AKT3* targeted by miR-326, thereby providing suppression of ErbB/PI3K pathway, detected by RT-qPCR, and dual luciferase assay. In addition, Western blot analysis revealed that miR-326 upregulation decreased PI3K signaling activity by decreasing total AKT and p-AKT protein level in SKBR3 cell lines. Interestingly, up regulation of ErbB2 rescued the effect of miR-326 on miR-326 target genes. Further functional assays demonstrated that up regulation of miR-326 significantly suppressed cell growth as evidenced by cell cycle, cell cycle associated genes expression, colony formation and MTT assays and induced apoptosis, detected by Annexin V-PI. In addition, EMT markers RT-qPCR, scratch, and Transwell assays showed inhibited cellular migration and invasion following miR-326 upregulation. Altogether, our results revealed that miR-326 play a tumor-suppressive role in breast cancer through inhibiting ErbB/PI3K pathway and miR-326 may serve as a potential therapeutic target for the treatment of patients with breast cancer.

## Introduction

Breast cancer is the most prevalent malignancy and the leading cause of cancer death in woman population worldwide (1). Genetic and epigenetic alterations of cell signaling pathways accompanied by considerable molecular and cellular heterogeneity represents one of the greatest challenges in variable prognosis and breast cancer treatment (2, 3). In spite of tremendous advances, the details and related mechanisms of breast cancer progression is still poorly understood. Therefore, elucidating the molecular underpinnings responsible for breast cancer development are crucially important to establish cutting-edge therapeutic strategies to prevention of this disease and to improvements in its diagnosis, prognosis, and treatment.

RETRACTED

ErbBs, typical receptor tyrosine kinases, comprise four members: EGFR /ErbB1/HER1, ErbB2/HER2, ErbB3/HER3, and ErbB4/HER4 (2). Activation of the ErbB family receptors (by homo- or heterodimerization) trigger two major downstream pathways, PI3K/AKT and MAPK (2). It has been shown that ErbB family members have important role in the initiation and maintenance of several solid tumors in which the HER2–HER3 heterodimer functions as an oncogenic factor by activating the PI3K/AKT signaling pathway (4, 5). Previous studies have reported deregulation of PI3K (in 70% of tumors) and MAPK (in 2–10% of tumors) pathways in breast cancer that could mediate resistance to anti-HER2 therapies and other anti-cancer agents (6–9). For this reason, ErbB receptors and major components of the PI3K and MAPK pathways are promising targets for breast cancer therapies and diagnosis (10). Hence, a better understanding of regulatory elements linking ErbB/PI3K signaling pathway could potentially propose strategies to prevent breast cancer.

MicroRNAs are a family of small non-coding RNAs with a short length of 19–25 nucleotides that function as oncogene or tumor suppressor by regulating a large number of protein-coding genes expression via mRNA degradation and translation blockage in a sequence-specific manner (11, 12). Recent progress in cancer biology has revealed the role of miRNAs in different physiological and pathological conditions (13) and abnormal expression of miRNAs is thought to contribute to the progression of cancers by regulating critical cancer-related genes and signaling pathways (14). But there is still large amount of unknown details that need to be explored further.

Several publications have appeared in recent years documenting various well-known miRNAs that affect ErbB/PI3K and MAPK signaling pathways and particularly some interesting microRNAs due to their importance in cancer development. For instance, miR-125a and miR-125b (15), miR-7 (16), miR-331-3p (17), and miR-21 (18) by suppressing different components can regulate PI3K signaling pathway and also have shown that miR-326 could be modulates MAPK/ERK signaling by regulating KRAS (19). Multi-level regulation of the signaling pathways by these miRNAs demonstrate their special ability in prognosis and cancer therapy.

RETRACTED

In the current study, by implementing bioinformatics and experimental approaches, we tried to find a microRNA that may play important role in regulating ErbB/PI3K signaling pathway. Using TCGA and GEO databases, we found miR-326 as a differentially expressed microRNA in breast cancer. Functional analysis suggests that miR-326 is a potential tumor suppressor that regulates ErbB/PI3K signaling by targeting a network of genes (*EGFR, ErbB2, ErbB3, AKT1, AKT2*, and *AKT3*) linked to these pathways and therefore, possibly controls breast cancer cell proliferation, EMT, migration, and invasion.

## Materials and Methods

### Bioinformatics Analysis

The microRNA expression data of breast cancer was retrieved from TCGA (https://tcga-data.nci.nih.gov/) NCBI and GEO (GSE40267/57897/19536/37407) (https://www.ncbi.nlm.nih.gov/geo/) databases. Potential target genes for miR-326 were predicted using TargetScan (http://www.targetscan.org/), miRanda (http://www.microrna.org/) and DIANA-microT-CDS online analysis tools (20–22). CLIP-seq data from Starbase v3.0 database (http://starbase.sysu.edu.cn/) was used for identifying the genes that directly interacts with miR-326 (23). Biological pathway analyses were performed by DAVID (https://david.ncifcrf.gov/) and DIANA-miRPath v3.0 (http://www.microrna.gr/miRPathv3) (24, 25).

### Cell Culture and Tissue Samples

Breast cancer tissues and adjacent normal breast tissues were obtained from Breast Cancer Research Center, Motamed Cancer Institute, ACECR, Tehran, Iran. All the tissue samples were collected, immediately snap frozen in liquid nitrogen, and stored at −80°C until RNA isolation. Informed consent was obtained from all patients.

The human breast cell lines, namely, SKBR3, MDA-MB-231, HS578T, and MCF7 were grown in HDMEM (Gibco), BT474 cells were grown in RPMI medium, and HEK293t cells were cultured in DMEM-F12 (Gibco) supplemented with 10% FBS(Gibco), penicillin (100 U/mL), and streptomycin (100 U/mL), which were maintained in a humidified incubator at 37°C with 5% CO_2_. All these cell lines were obtained from Pasteur Institute/Iran.

### Transfection

Complete medium without antibiotics was used to culture the cells at least 24 h prior to transfection. The cells were washed with PBS (pH 7.4) and then transiently transfected using Lipofectamine™ 2000 (Invitrogen) or TurboFect Reagent (Thermo Scientific) according to the manufacturer's instructions.

### RNA Extraction and Quantitative Real-Time PCR

Total RNA from the cultured cells and tissues was extracted using RiboX reagent (Invitrogen) according to the manufacturer's instructions. Extracted RNA was analyzed for its purity and integrity by spectrophotometry and gel electrophoresis. RNA (2 μg) was converted into cDNA using Reverse Transcriptase (Takara). For miRNA detection polyA tail was added to the 3′ end of RNAs before cDNA synthesis. QRT-PCR was performed using BIOFACT™ 2X Real-Time PCR Master Mix in the Applied Biosystems StepOne Real-Time PCR. GADPH and U48 were used as internal controls. The relative expression level was calculated using the 2^−ΔΔ*Ct*^ and 2^−Δ*Ct*^ methods. Primers and oligo sequences used in this study are listed in Supplementary Table 1.

RETRACTED

### Dual-Luciferase Reporter Assay

PsiCHECK-2 dual luciferase vector (Promega) was used to clone the 3′-UTR of all the predicted target genes of miR-326. To study direct interaction, HEK293T cells were co-transfected with wild-type (control) reporter plasmid (psi-check2 construct) and miR-326 (mock vector) using TurboFect Reagent (Thermo Scientific). A fragment with no predicted microRNA recognition element (MRE) for miR-326 was used as a control. **Forty-eight** hours after transfection using dual-glo luciferase reporter system, the activities of the Firefly and Renilla luciferases were measured sequentially from cell lysates, according to the manufacturer's instructions (Promega). Firefly luciferase units were normalized against Renilla luciferase units to control the transfection efficiency.

### Cell Cycle Assay (Flow Cytometry)

Cells were harvested 36 h after transfection and then centrifuged at 1,200 rpm for 5 min and washed twice in PBS. Subsequently, fixed with 500 μl of 70% cold ethanol for 2 h. The cells were added with 500 μl of PI/RNase staining solution and incubated at 37°C for 30 min away from light. The samples were immediately subjected to flow cytometer (BD, San Diego, CA, USA). The results were analyzed using FlowJo software (version10, TreeStar, USA).

### Apoptosis Assay

SKBR3 cells apoptosis was tested using Annexin V-FITC/PI staining kit according to the manufacturer's instruction (Roche, Germany). SKBR3 cells were cultured in 12-well plates with serum-containing complete medium. Thirty-six hours after transfection, the cells were washed with cold PBS and resuspended in binding buffer (100 mM HEPES, pH 7.4, 100 mM NaCl, and 25 mM CaCl2), followed by staining with Annexin V-FITC/PI at room temperature in the dark for 15 min. Apoptotic cells were then evaluated by gating the PI- and Annexin V-positive cells using a FACS flow cytometer (BD, San Diego, CA, USA). Data were subsequently analyzed by FlowJo software (version10, TreeStar, USA).

### Cell Proliferation Assay (MTT Assay)

SKBR3 cells were seeded as triplicate in 96-well plates and then were transfected with miR-326 or mock vectors. 24 and 48 h after transfection, the cells were treated with MTT to quantify the number of viable cells. Hence, 20 μl of MTT (5 mg/ml in PBS) was added to the cells. **Four** hours after MTT addition, the supernatant was discarded and the formazan crystals were dissolved in DMSO (100 μl). Subsequently, the absorbance at 570 nm was measured using a multi-well plate reader.

RETRACTED

### Colony-Formation Assay

SKBR3 cells (500 per well) were seeded in a six-well plate. After transfection, fresh media replaced every 2 days. After 10 days of culture, cells were fixed by ice-cold ethanol and stained with 1% crystal violet (40× and 100× magnification).

### Wound-Healing Assay

SKBR3 cells were seeded in a 24-well plate and incubated for 24 h. After transfection, a straight wound line was made by scraping with a sterile 20-μl pipette tip across the cell monolayer. Cells were washed with PBS and cultured in HDMEM supplemented with 10% FBS. The movement of cells toward the wound at different time points were captured under the microscope (40× magnification) and the images was analyzed with ImageJ (version 1.52a).

### Western Blot Assay

Thirty hours after transfection, SKBR3 cells were lysed in RIPA buffer, and protein concentrations were measured by Bradford assay. Total protein was separated by SDS-PAGE using a 10% polyacrylamide gel and electroblotted onto a PVDF. The membrane was immunoblotted overnight at 4°C with primary antibodies against phospho-AKT (Santa Cruz, USA, sc-514032), AKT (cell signaling), and β-actin (Santa Cruz, USA, sc-130301) and a secondary goat anti-mouse antibody (BIORAD, USA, 1721011) were diluted according to the manufacturers' instructions and was incubated with the membrane for 1 h after three washes with TBST. Signals were detected with ECL detection reagent (Pierce, Rockford, IL). The images were obtained by Quantity One (Bio-Rad). Original blots are shown in Supplementary Figure 1.

### Transwell Assay

Migration and invasion assays were performed using a Transwell system (8-μm pore size; Corning Inc., Corning, NY, USA). For the migration assay, 5 × 10^5^ cells were seeded in the upper chamber. For the invasion assay, the membrane was coated with Matrigel to form a matrix barrier, and 4 × 10^5^ cells were placed in the upper chamber in serum deprived culture (DMEM supplemented with 1% FBS). In each lower chamber, serum-free medium with 10% FBS was added. After 24 h incubation at 37°C, cells that had migrated through the pores were fixed and stained with 0.1% crystal violet solution, washed with PBS, and photographed.

### Statistical Analysis

All experiments were performed in triplicates independently. The results are presented as the means ± standard error mean (SEM). The *t*-test or One-Way Analysis of Variance (ANOVA) was performed using GraphPad Prism software in order to determine significant differences in measured variables among groups. *P*-value < 0.05 was considered as statistically significant.

RETRACTED

## Results

### Hsa-miR-326 Is Aberrantly Down-Regulated in Human Breast Tissues and Cell Lines and Correlated With Poor Prognosis

To confirm that our microRNA was differentially expressed in breast cancer and acts as a tumor suppressor through regulation of the ErbB/PI3K pathway, TCGA cohort, and multiple GSE dataset analysis were performed accompanied by target prediction software and CLIPseq data analysis. Eventually, bioinformatics suggesting that miR-326 could have important functions in breast cancer through regulating ErbB/PI3K pathway, therefore it was selected for further investigation (Figure 1A).

**Figure 1:** Expression of miR-326 in human cancerous and normal breast tissues and cell lines. **(A)** miR-326 selection strategy flowchart **(B)** Differential expression of miR-326 in breast cancer and non-cancerous tissues from the TCGA database. **(C)** Expression profiles of miR-326 in breast cancer and normal breast tissues, in breast cancer patients with low proliferative (LP) and high proliferative (HP) tumors and in primary and metastatic tumors from (GSE57897, GSE19536, and GSE37407) datasets, respectively. **(D)** Kaplan–Meier survival analysis of breast cancer patients from GSE40267 dataset with different miR-326 expression. **(E)** The miR-326 expression in human breast cancer tissues compared to their adjacent normal pairs were detected by RT-qPCR. *N* = 20 for each group. **(F)** The mean Fold Change for breast cancer patient. **(G)** ROC curve for identification of patients with breast cancer vs. healthy controls (*N* = 20 for each group) using miR-326. AUC, area under the ROC curve. **(H)** Expression of miR-326 in aggressive and less-aggressive breast cancer cell lines from GSE40059 dataset. **(I)** The mean of expression for each group. **(J)** RT-qPCR analysis of the miR-326 in aggressive and less- aggressive breast cancer cell lines. Assays were performed in triplicate. Means ± SEM was shown. Statistical analysis was conducted using student *t-*test.

To determine whether miR-326 was differentially expressed in breast cancer patients and correlated with tumor formation and metastasis, RNA seq (adopted from TCGA) and array data (adopted from GEO) were analyzed. In the TCGA cohort, miR-326 expression was decreased in the 1,085 BRCA (breast invasive carcinoma) tissues compared to 104 normal breast tissues (*p*-value = 9.3e-17, Figure 1B). Also, analysis of multiple miRNA expression profiling array data set have demonstrated that miR-326 was significantly down-regulated in 419 breast cancer tissues compared to 31 normal breast tissues (*p*-value = 0.0498, GSE57897). Furthermore, low expression of miR-326 was observed in 37 high proliferative tumors compared to 64 low proliferative ones (*p*-value = 0.0045, GSE19536). Additionally, the expression of miR-326 significantly decreased in 17 primary tumors with respect to 31 metastatic samples (*p*-value = 0.0045, GSE37407, Figure 1C).

RETRACTED

To examine the association of miR-326 with clinic-pathological features of breast cancer patients, Kaplan-Meier analysis was evaluated. These patients were categorized into patients at high/low-risk groups based on the expression levels of the miRNA and revealed that the BRCA patients with low miR-326 levels had worse overall survival time when compared with patients with high expression levels of this microRNA (log-rank test: *p*-value = 0.01, GSE40267, Figure 1D).

To verify the suppression of miR-326 in breast cancer specimens, the mature miR-326 expression level was measured using RT-qPCR. The results indicated that miR-326 expression was strongly down-regulated (mean ~50% reduced) in 20 breast cancer specimens in comparison with matched-normal tissues (*p*-value < 0.001, Figures 1E,F).

To examine the power of miR-326 in breast cancer detection, ROC curve was used to evaluate the sensitivity and specificity of miR-326 expression level for discrimination of breast cancer specimens vs. non-tumor samples. The area under curve (AUC) of miR-326 was evaluated 0.72 (*p*-value = 0.01, Figure 1G), which is a score more than the cutoff (0.7) needed for a considerable biomarker.

Bioinformatics analysis of miR-326 expression in GSE40059 dataset showed significantly lower levels of miR-326 in aggressive breast cancer cell lines compared to less aggressive (*p*-value < 0.05, Figures 1H,I). In consistent with bioinformatics data, RT-qPCR result revealed that the aggressive breast cancer cell lines including, MDA-MB-231 and HS578T expressed a lower level of miR-326, relative to that of less aggressive breast cells BT474, MCF7, and SKBR3 cells. The data indicate that the cells with more aggressive characteristics have lower expression of this microRNA (Figure 1J).

Altogether, these results show that miR-326 expression decreases in cancerous breast tissues with respect to normal one and also its expression in more aggressive cell line is lower. Furthermore, miR-326 expression is negatively correlated with tumor proliferation and aggressiveness and the patients with low levels of miR-326 expression have poor survival rate. Additionally, the miRNA can discriminate BRCA patients with relatively high accuracy and could be valuable biomarker for BRCA detection. Therefore, our data suggest that miR-326 may act as a tumor suppressor factor in breast cancer.

RETRACTED

### Hsa-miR-326 Targets a Gene Network in ErbB/PI3K Pathway

In order to identify target genes of miR-326 in ErbB/PI3K pathway, several computational miRNA target prediction tools (TargetScan, miRanda and DIANA-microT-CDS) have provided putative binding sites for this miRNA. As shown in (Table 1), there were best complementary pattern of the miR-326 and 3′-UTRs of the ErbB2, ErbB3, AKT1, AKT2, and AKT3 mRNAs. Furthermore, CLIP-seq data retrieved from StarBase v3.0 was used to identify the genes that may directly interacts with miR-326 (Table 2). Argonaute CLIP-Seq data reveals the miRNA-target interactions through intersecting the predicting target sites of miRNAs with binding sites of Argonaute protein.

**Table 1:** Transcript position and seed sequence of miR-326 on the 3′UTRs of *ErbB2, ErbB3, AKT1, AKT2*, and *AKT3* genes (the best scored alignments were shown in the table).

**Transcript position**	**Alignment**
314–320	
861–876	
384–411	
1,321–1,338	
778–784	

**Table 2:** CLIP-seq data indicated interaction of MiR-326 with *EGFR, ErbB2, ErbB3*, and *AKT2* genes adopted from Starbase v3.0.

**Genes**	**Bincling site**	**RBP**	**Seq type**	**Cell/Tissue**	**Accession**
*EGFR*	chr7:55273756-55273800[+]	AG02	HITS-CLIP	HeIa	GSM1048187
*ErbB2*	chr17:37384260-37884305[+]	AG02	HITS-CLIP	HeIa	GSM1048186
*ErbB3*	chr12:56495777-56496127[+] chr12:56495810-56495879[+]	AG01-4 AG01-4	HITS-CLIP HITS-CLIP	MCF7 Liver	GSM2065792 GSE97056
*AKT2*	chr19:40739848-4074 099 6[–]	AG02	AR.C:L P	DG75-BCBL-1	GSE43909

To confirm the effect of miR-326 on ErbB/PI3K signaling pathway genes, the changes in their expression in SKBR3 cells upon miR-326 overexpression was examined. EGFR, ErbB2, ErbB3, AKT1, AKT2, and AKT3 significantly decreased at the mRNA expression level in SKBR3 cells over-expressing miR-326 compared to mock transfected cells (*p*-value < 0.05, 0.01, 0.05, 0.01, 0.05, and 0.05, respectively, Figure 2A). To investigate the direct interaction of ErbB2, ErbB3, AKT1, and AKT2 with miR-326, dual luciferase reporter assay was performed. For this reason, the 3′-UTR of each target gene have been cloned downstream of the Renilla luciferase gene. Luciferase activity of ErbB2, ErbB3, AKT1, and AKT2 in HEK293 was decreased after co-transfection of 3′-UTR with miR-326 relative to the mock and No-MRE control (a plasmid lacking any binding site for the miRNA) vectors (*p*-value < 0.05, 0.01, 0.05, and 0.01, respectively, Figure 2B). Furthermore, western blot analysis confirmed the reduction at the phospho-AKT and total AKT protein level after miR-326 overexpression compared to mock transfected cells (*p*-value < 0.01, Figure 2C).

RETRACTED

**Figure 2:** miR-326 targets multiple genes in ErbB/PI3K pathway. **(A)** RT-qPCR results of the expression of potential targets (EGFR, ErbB2, ErbB3, AKT1, AKT2, and AKT3) upon miR-326 and mock vectors transfection in SKBR3 cells. **(B)** Relative luciferase activity of reporter plasmids carrying the wild-type UTR or a fragment lacking any binding site for miR-326 (as a control UTR) in HEK293 cells co-transfected with miR-326 or mock vector. **(C)** Expression level of phospho-Akt and total AKT protein were detected by Western blotting in miR-326 and mock transfected SKBR3 cells. **(D)** ErbB2, ErbB3, and AKT1 expression levels in SKBR3 cells transfected with ErbB2 psicheck or co-transfected with ErbB2 psicheck and mock or miR-326 were significantly higher than the cells transfected with control vectors (mock, psicheck empty vector, and combination of mock and psicheck vectors) that indicates ErbB2 rescued miR-326 target genes (ErbB2, ErbB3, and AKT1 genes). In contrast, ErbB2, ErbB3, and AKT1 expression levels in SKBR3 cells transfected with miR-326 or co-transfected with psicheck empty vector and miR-326 were significantly lower than the cells transfected with control vectors (mock and combination of mock and psicheck vectors). Assays were performed in triplicate. Means ± SEM was shown. Statistical analysis was conducted using student *t*-test.

Moreover, to elucidate whether up-regulation of miR-326 target gene could rescue the effects of miR-326 on other target genes, we investigated ErbB2 psicheck overexpression effect on miR-326 target genes by RT-qPCR. ErbB2, ErbB3, and AKT1 expression levels in SKBR3 cells transfected with ErbB2 psicheck or co-transfected with ErbB2 psicheck and mock or miR-326 were significantly higher than the cells transfected with control vectors (mock, psicheck empty vector and combination of mock and psicheck vectors) that indicates ErbB2 rescued miR-326 target genes (ErbB2, ErbB3, and AKT1 genes). In contrast, ErbB2, ErbB3, and AKT1 expression levels in SKBR3 cells transfected with miR-326 or co-transfected with psicheck empty vector and miR-326 were significantly lower than the cells transfected with control vectors (mock and combination of mock and psicheck vectors; Figure 2D).

Taken as a whole, these approaches confirmed that miR-326 can regulate ErbB/PI3K pathway through targeting the mentioned genes.

### Hsa-miR-326 Suppresses Breast Cancer Cell Proliferation and Promotes Apoptosis

The inhibitory role of miR326 on SKBR3 breast cancer cell proliferation was investigated by cell cycle analysis, cell cycle genes expression, and colony formation assay. Cell cycle analysis revealed that overexpression of miR-326 compared to mock and scrambled transfected cells, resulted in a considerable increase of the sub-G1 cell proportion and a decrease in the G0/G1, S, and G2/M cell proportions (*p*-value < 0.0001, Figures 3A,B). Furthermore, to study the effect of miR-326 on the expression level of cell cycle-associated genes, *Cyclin D1* and *Cyclin D2* (components of the core cell cycle machinery) gene expression were examined. The results showed that miR-326 decreased the mRNA expression level of cyclin D1 and cyclin D2 (*p*-value < 0.01, Figure 3C) in SKBR3 cells overexpressing miR-326 compared to mock transfected cells. Additionally, overexpression of miR-326 remarkably inhibited colony formation in SKBR3 cells compared to mock transfected cells (40× and 100× magnifications, Figure 3D). Altogether, these results show that miR-326 suppresses cell growth in SKBR3 cells.

RETRACTED

**Figure 3:** Effects of miR-326 overexpression on cell cycle, proliferation, and apoptosis of SKBR3 cells. Histogram **(A)** and bar plot **(B)** analysis of SKBR3 cell cycle transfected with either miR-326 overexpressing or mock or scrambled vectors, 36 h after transfection. **(C)** Expression of CCND1 and CCND2 in transfected SKBR3 cells. **(D)** Represents photomicrographs of colony formation assay of SKBR3 cells after transfection with miR-326 and mock vector for 10 days (40× and 100× magnification). **(E)** MTT assays of SKBR3 cells after transfection with miR-326 or mock vector. **(F,G)** Cell apoptosis assay was performed to determine the apoptosis rate following transfection of miR-326, mock, and scrambled vectors, Histogram **(F)** and bar plot **(G)** of cell percentage in each phase **(H)** Expression of Bcl-2, Bcl-XL, and Bax mRNA in SKBR3 cells after transfection with miR-326. Assays were performed in triplicate. Means ± SEM was shown. Statistical analysis was conducted using student *t*-test and one-way ANOVA.

To further validate the anticancer role of miR-326 in breast cancer, its effect on breast cancer cell (SKBR3) viability was investigated using MTT assay. The results demonstrated that miR-326 over-expression significantly attenuated SKBR3 cells viability at 24 and 48 h after transfection (*p*-value < 0.001, Figure 3E).

Due to the noticeable increase in the sub-G1 phase, the role of miR-326 on SKBR3 cells apoptosis was evaluated by PI/Annexin V assay and apoptotic and anti-apoptotic genes expression. The results of flow cytometric analysis demonstrated that overexpression of miR-326 resulted in a remarkable increase in late apoptotic cells of SKBR3 with respect to the mock and scrambled transfected cells (*p*-value < 0.0001, Figures 3F,G). Furthermore, miR-326 also inhibited the expression level of anti-apoptotic Bcl2 and Bcl-XL and significantly increased expression level of Bax mRNA (*p*-value <0.05, 0.01, and 0.05, Figure 3H). These results demonstrated that miR-326 indeed promoted apoptosis in SKBR3 cells.

RETRACTED

### Hsa-miR-326 Inhibits Breast Cancer Cell Migration and Invasion

To assess the role of miR-326 on SKBR3 cells migration and invasion, as characteristics of metastatic cancer cells, three different approaches were performed. Firstly, wound healing assay was used. Migration of cells at different time points (0, 12, 24, 36, 48 h) after scratching was monitored under a microscope. Relative ratios of wound closures in SKBR3 mock transfected cells was significantly more than miR-326-expressing cells after 36 and 48 h of transfection (*p*-value < 0.05, Figures 4A,B).

**Figure 4:** Effects of miR-326 overexpression on cell migration and invasion. **(A)** A wound healing assay in SKBR3 cells transfected with either miR-326 or mock vector at 0, 12, 24, 36, and 48 h post-scratching (40× magnification) **(B)** Quantitative analysis of scratch wound closure **(C)** RT-qPCR showing the expression of epithelial and mesenchymal markers in SKBR3 cell lines upon miR-326 transfection compared to mock vector transfected cells. **(D)** Transwell migration and invasion assays after transfection of SKBR3 cells with miR-326 or mock vectors. Assays were performed in triplicate. Means ± SEM was shown. Statistical analysis was conducted using student *t*-test.

Secondly, to assess miR-326 effect on epithelial to mesenchymal transition (has been proposed as a key process in cancer progression), *Claudin1* (epithelial marker), *ZEB1, Snail, Twist2*, and *B-catenin* (mesenchymal markers) genes expression were checked in SKBR3 cells. An increase in the expression of epithelial marker (*p*-value <0.05) and a decrease in expression of Snail, Twist2, and B-catenin mesenchymal markers (*p*-value < 0.05, 0.01, and 0.05, respectively) indicated that restoring the expression of miR-326 reduced breast cancer invasive capacity. But the decline in ZEB1 expression was not observed (Figure 4C). In the third approach, to investigate the role of miR-326 on SKBR3 cells migration and invasion, Transwell assay was used. In the migration assay, miR-326 transfected cells showed a decreased migratory ability compared to mock transfected cells. Similarly, in the invasion assay, miR-326 transfected cells showed a decrease in the ability to traverse though the matrigel-coated membrane (*p*-value < 0.01; Figure 4D).

RETRACTED

These results, taken together, represented that miR-326 expression importantly reduces the migration and invasion mobility of breast cancer cells.

## Discussion

Breast cancer is one of the most prevalent malignancy in women worldwide (1) and increasing evidence have demonstrated the importance of ErbB/PI3K pathway in breast cancer tumorgenesis (26–28). ErbB receptors and protein kinases located along this pathway represent very attractive and promising drug targets for anticancer therapies. Hence, understanding the molecular mechanism of ErbB/PI3K deregulation and finding the regulators of this pathway could be beneficial for future cancer research and also cancer prevention and treatment. Recent studies have shown that microRNAs, as a layer of gene regulators, can regulate ErbB/PI3K pathway through targeting numerous target genes and play important role in cancer progression (29).

To find a microRNA that may play critical role in breast cancer, RNA sequencing and array data accompanied by target prediction tools and CLIP-seq data were evaluated. Based on several bioinformatics analyses miR-326 selected for further research, suggesting that there may be some critical link between miR-326 and breast cancer. It has been shown that miR-326 is negatively correlated with MRP-1 expression in breast cancer and may be an efficient agent for multi-drug resistance (30). However, the underlying mechanism of action of miR-326 through ErbB/PI3K signaling pathway in breast cancer is poorly studied. The aim of this study is investigating miR-326 function as potential tumor suppressor gene in modulating ErbB/PI3K pathway in breast cancer progression.

Although individual miRNAs can have either oncogenic or tumor-suppressive function, several reports have indicated widespread disruption of miRNA expression levels in numerous cancers (12, 13). Also, substantial evidence has shown that some deregulated miRNAs can be used as prognostic biomarkers as well as powerful therapeutic targets in breast cancer (31–33). Our bioinformatics and experimental analysis have identified miR-326 as a miRNA that aberrantly expresses in breast cancer tissues and cell lines. The altered expression of miR-326 in cancerous tissues and cell lines establishing the functional importance of the observed down-regulation of candidate microRNA in tumors and supporting the potential utility of these miRNAs to monitor BRCA patients and highlighting their clinical value for breast cancer detection and surveillance. Subsequently, the low expression level of miR-326 positively associated with tumor proliferation, metastasis, and poor survival. Our findings are largely in accordance with the previous studies for a number of malignancies, including colorectal (34), hepatocellular (35), glioma (36), glioblastoma (37), osteosarcoma (38), and non-small cell lung cancer(NSCLC) (39), which in these studies miR-326 is down-regulated and possibly acts as a tumor suppressor.

RETRACTED

Currently, numerous small molecular drugs that inhibit ErbB receptors, PI3K, AKT, and/or mTOR are being developed in preclinical and clinical models of breast cancer (40–44). In our present study, we are trying to introduce an endogenous regulator of the ErbB/PI3K pathway. The bioinformatics data and experimental approach show that miR-326 controls expression of ErbB/PI3K signaling genes in transcriptional and translational level by modulating the genes involved in the pathway and therefore changes the expression of downstream target genes involved in cell cycle and apoptosis regulation. In addition, up regulation of ErbB2 rescued the effect of miR-326 on other predicted target genes. Thus, these results support the idea that miR-326 mediates its tumor suppressive effects, at least in part, through direct or indirect targeting and functionally inhibiting these key genes of ErbB/PI3K pathway.

Multiple studies supporting the role of ErbB/PI3K in cell cycle and apoptosis regulation by modulating the downstream genes involved in these pathways (45–47). For instance, *Akt*, as a bottleneck gene of this pathway, triggers a network that positively regulates cell cycle progression and also suppresses programmed cell death (48, 49). To further explore the putative tumor suppressive function of miR-326 in human breast cancer cell lines, the mechanism of miR-326 on the cell growth and viability in SKBR3 cell lines was examined, and found that overexpression of miR-326 significantly inhibited cell proliferation as evidenced by cell cycle, cell cycle associated genes expression, colony formation, and MTT assays. Remarkably, another study demonstrated that CCND1, which plays a critical role in promoting G1–S transition, was recently identified as a direct target of miR-326 (39, 50). Therefore, the growth-inhibition role of miR-326 may attribute to inhibition of ErbB/PI3K and cyclin D1 expressions. In addition to inhibition of cell proliferation, the growth inhibitory effect of miR-326 was also related to induction of apoptosis detected by Annexin/PI assay and through the measurement of the apoptotic and anti-apoptotic gene expression. Also, previous studies reported that miR-326 targets Bcl-2 (38) and Bcl-xL (51) and thereby mediating apoptosis. Hence, miR-326 by targeting ErbB/PI3K and apoptosis-related genes can regulate cell death directly or indirectly.

RETRACTED

EMT is accompanied by alterations in cell morphology, cell-cell adhesion, the activity of cellular signaling pathways, and the extracellular matrix. Therefore, tumor cells are capable of invasion into the surrounding environment and eventually distant sites through blood and lymph (52). ErbB/PI3K signaling has been described as one of the important factors through the regulation of epithelial-to-mesenchymal transition and the transcriptional control of metastasis-related genes (53, 54). In this study, EMT-involved genes expression, migration, and invasion capacity of breast cancer cells decreased upon miR-326 overexpression, which suggest that this miRNA may also function as a metastasis suppressor by blocking these pathways.

Taken together, our results demonstrated that miR-326 expression was down-regulated in breast cancer and this low expression was correlated with the tumor proliferation, metastasis, and poor prognosis of breast cancer patients. Our findings would seem to indicate that miR-326 is a regulator of cell proliferation, apoptosis, migration and invasion in breast cancer through targeting a gene network of ErbB/PI3K pathway (Figure 5), suggesting that miR-326 may serve as a promising target and diagnostic marker for treating breast cancer in the future. Although, these findings are promising, further data collection would be needed to determine exactly how miR-326 is down-regulated and affects breast cancer.

**Figure 5:** Schematic representation of ErbB/PI3K pathway regulation by miR-326. In this model, miR-326 by targeting the ErbB2, ErbB3, and AKT transcripts, results in reduced PI3K signaling pathway activity which in turn, affects the biological process of cells, including proliferation, apoptosis, invasion, and migration.

## Ethics Statement

Informed consent was obtained from all patients.

## Author Contributions

ZG: Performed the experiments and analyzed data and wrote manuscript. ZG and BS: Designed experiments. BS: Supervised the study. SM: Advised the research.

### Conflict of Interest Statement

The authors declare that the research was conducted in the absence of any commercial or financial relationships that could be construed as a potential conflict of interest.
